The article "Feedforward Control Combined with 4F Management on Postoperative Nursing Effects and Motor Function of Meniscus Sports Injuries: Based on a Prospective Case Analysis" was retracted in 2023. Reasons: unreliable results or conclusions; lack of ethics approval or compliance; concerns about the data; concerns about the peer review.

# Feedforward Control Combined with 4F Management on Postoperative Nursing Effects and Motor Function of Meniscus Sports Injuries: Based on a Prospective Case Analysis

**DOI:** 10.1155/2022/5447509

**Published:** 2022-07-09

**Authors:** Qin Lu, Qunya Yu

**Affiliations:** ^1^Department of Pediatrics, Shanghai Jiao Tong University Affiliated Sixth People's Hospital, Shanghai 201306, China; ^2^Department of General Surgery, Shanghai Jiao Tong University Affiliated Sixth People's Hospital, Shanghai 201306, China

## Abstract

**Background:**

Because active functional training and management after knee cartilage sports injury is the key to treatment, care of patients after an operation with knee cartilage sports injury is critical.

**Aims:**

To explore the effect of feedforward control combined with 4F management and after an operation nursing effect on patients with knee cartilage sports injury.

**Materials and Methods:**

According to the random number table method, 100 patients with knee cartilage sports injury who were nursed in our hospital from June 2019 to June 2021 were selected as the research objects and divided into the control group and the instance of watching, noticing, or making a statement group with 50 cases in each group according to the different nursing order. Among them, the control group adopted 4F management combined with feedforward control nursing mode: all-weather, whole-process, whole-system, and all-around services for patients. On this basis, the instance of watching, noticing, or making a statement group cooperated with early healing/repairing training to compare fear and stress-related self-test of the two groups of patients after an operation. Knee function and quality of care are scored using tables.

**Results:**

After nursing, the knee joint function score of the instance of watching, noticing, or making a statement group was higher than that of the control group, while the pain after the operation, sleep quality, fear, and stress self-rating scale scores were significantly lower than the control group (*P* < 0.05). The whole-process management, body position placement, risk evaluation, repairing training, all-weather service, whole-system management, and comprehensive service of the two groups of patients were very much improved. The nursing quality of watching, noticing, or making a statement group was significantly higher than the control group (*P* < 0.05).

**Conclusion:**

Feedforward control combined with 4F management combined with early repairing training can effectively reduce the fear and stress after an operation pain and sleep quality of knee cartilage sports injury and help increase the recovery of knee combined function in a good way.

## 1. Introduction

With the fast development of a social process of people making, selling, and buying things and the gradual moving ahead or up of growth of cities with more people, the number of times something happens of breaks caused by violent injuries such as falls from heights and car crashes is increasing, and knee cartilage sports injuries are more common [1]. As a more common type of joint injury in the clinic, physical labor and excessive exercise are the main factors causing knee injury [2]. After knee injuries, most of them are accompanied by multiple structural and functional injuries. The degree of pain is severe, the patient's normal activities are restricted, and the knee joint is swollen and unable to straighten, which seriously affects the quality of life of patients [3].

The knee cartilage is embedded between the lower-leg bone condyle and the inner and outer condyles of the thigh bone. Its function is to prevent friction, reduce shock, spread synovial fluid, moisten the joint, and soak it up like a towel heater. Meniscal injury is a common disease of the knee joint [4]. Clinically, surgery is often used to treat meniscal injuries, such as meniscus plasty, meniscus repair and suturing, and meniscal subtotal resection, which was more common in the past two. Surgical treatment can greatly improve the patient's clinical symptoms and improve the quality of life of the patient [5].

After knee cartilage sports injury, effectively early scrape away dead skin and break compound constant, and obsessive thoughts are performed through surgery. However, different degrees of knee joint mobility limitation, muscle strength decline, swelling, pain, and other functional sicknesses are usually left after the operation, which affects the after operation function of the patient. Recovery and medically beneficial effects can be seen in [6]. In addition, some patients will have complications such as pain after surgery, which seriously affects the recovery prognosis of patients. Therefore, more emphasis is placed on the prevention of postoperative pain in the clinic to promote patient recovery and improve prognosis. How to solve the difficulties of the knee combined harmful after an operation and angry behaviors and improve the quality of life of patients have become very hard research topics in the field of orthopedics [7]. Knee cartilage sports injury is a typical knee injury that leads to the destruction of the uninterrupted, constant quality and honest and good human quality/wholeness or completeness of the knee cartilage for different reasons often treated by surgery [8]. Because of active functional training and management after (knee cartilage sports injury is the key to treatment after an operation), care of patients with knee cartilage sports injury is especially important [9].

The 4F management model provides patients with all-weather, whole-process, whole-system, and all-around nursing services. Through careful, clean, and scientific nursing, the mental pressure of patients during the long-term healing/repairing process after surgery is relieved [10]. It can effectively solve the problems of patients in the process of healing, improve patients' trust in nurses, and help increase in a good way repairing [11]. Feedforward control refers to guessing a number of the results that can be produced before certain nursing care starts and taking the corresponding action that helps a bad situation measures for some unsafe factors before nursing in the 4F management model, which plays a role in preventing problems but does not have functional healing/repairing training [12]. Early functional repairing training can effectively improve the patient is not able to be harmed and able to get a disease and complete and thorough body structure, improve the muscle strength around the knee combined, help increase in a good way blood circulation, and speed up the recovery process of the body (following the law as you are told, improving the overall recovery of patients). 4F management on the basis of understanding the patient's physical, emotional, social, and cognitive functions analyzes the current situation and then carries out targeted nursing, in the event of a situation can be timely treatment [13]. Feedforward control refers to the use of data consulting, collecting data and information, mastering the rules, combined with the actual situation, estimating the possible problems of an operation, and taking preventive measures in advance to nip the risk factors in the bud [14]. The combination can not only avoid or mitigate the adverse effects of risk factors on patient treatment and prognosis on the basis of individualized care, thereby improving nursing safety [15]. Therefore, this study carefully studied the nursing effect of feedforward control combined with 4F management and early healing training on patients with knee cartilage sports injury after an operation and referred to medicine-based nursing of knee cartilage sports injury.

## 2. Material and Methods

### 2.1. Research Object

This study has been informed to patients and their families, signed based on knowledge and learning permission, and approved by the medical related to the rules and beliefs of doing the right thing group of our hospital. According to the random number table method, 100 patients with sports injuries of the knee cartilage in our hospital were selected as the research objects. According to the different nursing orders, they were divided into the control group and the instance of watching, noticing, or making a statement group with 50 cases in each group, including 37 cases of middle part knee cartilage injury and 50 cases of lateral knee cartilage injury. Injuries happened in 35 cases, and discoid knee cartilage in 28 cases. All knee cartilage sutures and partial or total meniscectomy were completed under arthroscopy. One hundred patients were randomly divided into an instance of watching, noticing, or making a statement group and a control group. The two groups of patients were compared in terms of age, female status, degree of injury, and other indicators, and there was no big difference (*P* > 0.05), which was similar.

### 2.2. Disease-Identifying Judging Requirements

The disease-identifying judging requirements for knee cartilage sports injuries go along with the disease-identifying judging requirements for meniscal sports injuries in the guidelines for the identification of a disease or problem or its cause and Treatment of Painful joint swelling (2018 Edition) [16]. Pain, swelling, combined snapping, and joint locking were the main visible signs, and the knee cartilage sports injury was identified disease or its cause by medicine-based and imaging studies. Suspected cases were judged by two orthopedic doctors that operate on people. In order to avoid bias in the judgment process, if the results of the two doctors were different, an agreement should be reached after discussion to decide/figure out whether there was a knee cartilage sports injury.

### 2.3. Exclusion Criteria

Inclusion criteria are as follows: (1) MRI and surgery confirmed all meniscus sports injuries, and the research subjects were ≥18 years old; (2) the patients had a certain ability of writing and language expression; (3) there was no joint, muscle damage, etc.; (4) voluntary participation; (5) complete clinical data are available.

Exclusion criteria as follows: (1) nonmeniscal sports injury; (2) selected patients without informed consent; (3) patients with severe mental illness, congenital, developmental, chronic organic diseases, and other trauma patients with secondary joint deformities and pain; (4) easy allergy to contrast agents; (5) malignancy, lactation or pregnancy, hematopoietic system disorders, and patients who cannot be complained about; and (6) concomitant disease of other lower extremity fractures.

### 2.4. Nursing Intervention Methods

#### 2.4.1. 4F Management

1. *All-Weather*. Set up a special green channel to ensure that patients receive the fastest care in the shortest time in the event of a sudden unplanned bad event. Answer or supervise patients to slowly complete functional exercises through WeChat groups or department telephones at any time to accomplish or gain with effort round-the-clock service. Any mental or physical problems that cannot be settled at home after the patient was released from hospital can be given the fastest help and support by specialist nurses
2. *The Whole Process*. This includes after an operation follow-up, after an operation serving to stop something bad before it happens, measures and self-management points, and after an operation mental change to make better to changing something. If there is no discomfort after the operation, the patient should drink water 2 hours after the operation and eat orally 4 hours after the operation
3. *Whole System*. Each patient is included in information management, and well-thought-out management is carried out according to the medicine-based path of surgery, including the form of the nurse's medicine-based path and the form of the patient's medicine-based path. At the same time, QQ groups are established to carry out sports injury health education through mobile networks
4. *All-Round*. After the act of letting someone enter/speaking the truth about something bad, a specialist nurse manages and does one-to-one interviews to understand the patient's thinking-related, feeling of love, hate, guilt, etc., social function, and family function. Provide targeted mental, physical, and social guidance, including appropriately timed management of after-drugs that cause numbness or unconsciousness difficulties. Nurses are responsible for health education, patiently explaining the steps taken to prevent trouble or injury, self-management knowledge of injury repair after discharge, and paying attention to the skin color, temperature, and swelling of the affected limb. On the second day after the operation, straight, lateral, and rear leg lifts were performed, and on the third day, active and allowing something to happen without reacting or trying to stop it, knee flexion exercises were performed, and the knee flexion angle slowly increased

#### 2.4.2. Feedforward Control Nursing Mode

(1) Establish a team: establish a dedicated feedforward control nursing team headed by the head nurse, organize nursing staff with different qualifications and educational backgrounds to carry out nursing management training, and change the nursing staff's idea of knee cartilage sports injury risk management. (2) Job management: the head nurse regularly manages and does on-the-job training for the nursing staff in the department and figures out the worth, amount, or quality of the effect. Strictly put into use the shift system, careful examination of something system, graded nursing system, and extremely sick patient rescue system, and clear up the responsibilities of each class. (3) Plan risk management plans: through regular ward rounds and monthly evaluations, nurses' risk knowledge about something and anti-risk ability has been made better. Identify possible problems in daily work such as whether the patient has pressure open, painful sores, and pain, figure out goals, plan plans, put into use effective measures appropriately timed change sheets and covers, pay attention toward the state of being clean, encourage patients to get out of bed, etc., and give reactions or responses to something/helpful returned information, through feedforward control for describing a possible future eventive and targeted management can reduce sudden unplanned bad crashes.(4) Nurse-patient communication: help patients establish a correct understanding of knee cartilage sports injury. Change the way of life, help increase the good way the patient faces the disease with a positive point of view, and actively cooperate with the treatment

### 2.5. Early Repairing Exercises

On the day of the operation, after the patient is awake from drugs that cause numbness or unconsciousness, instruct the patient to lie on the bed or stand, straighten the unaffected limb and push the heel back with force, 10~15 min, 1~2 times, forcefully tighten the quads of the thigh muscle, hold for 10 s, relax for 5 s, and repeat, 30 times/d. Two to 7 days after the operation, based on quadriceps training, add ankle flexion and extension training and knee combined booster lower limb straightening training, 10-15 min/time, 2-3 times/d. On the 8th to 12th day after the operation, added trainings such as straight leg raising, bedside knee flexion and extension, hip flexion and hip flexion, and active and allowing something to happen without reacting or trying to stop it exercise in the lying position were added, 10 to 15 min/time, 2 to 3 times/d. 13 days after the operation, the patient was released from hospital, and instruct the patient to increase resistance exercise, tie a sandbag on the patient's calf, the weight of the sandbag should be selected according to the patient's body, age, and pain level, and do back extension and forward flexion exercise training with the help of family members, 6 times, 2~3 times/d. Patiently explain the pain machine, causes, and steps taken to prevent trouble or injury to patients and their families, and give appropriate mental counseling to patients with fear, stress, and depression. For patients with a VAS score lower than 7 points, drug action that helps a bad situation measures was given to them, and limb massage combined with salt water cold bag cold cloth pressed against the skin on the tissues or other parts of the knee combined break/crack, 15 min, 2~3 times, instruct them to choose listening quick and energetic music, reading newspapers, and talking with friends or family members at all times to change to focus on or point at, a different direction of their attention from pain, add painkillers for patients with scores 7-10, and instruct patients to take reasonable painkillers as prescribed by the doctor.

### 2.6. Observation Indicators

There was no dropout or withdrawal during the 6-month follow-up in this study. The scores of the self-rating anxiety scale, Lysholm knee function score, and nursing quality were observed in the follow-up patients. ① Anxiety self-rating scale score below 50 is normal. The lower the score is, the less anxious the patient is. ② The Lysholm knee joint function score includes 8 aspects, scored from 0 to 100. The higher the score, the more the patient's knee meniscus motility, and the better the injury recovery. ③ The nursing quality assessment is jointly completed by all members of the nursing team, mainly assessing all-weather service, whole-process management, whole-system management, all-round service, rehabilitation training nursing, risk assessment, and postural placement, with a total of 10 points, the higher the score. High indicates better quality of care. The evaluation time was randomly selected three times in total, and the average value was taken. ④ VAS evaluates the pain of the two groups of patients through VAS. The evaluation standard is less than 3 points for mild pain, 4-6 points for pain affecting sleep, and 7-10 points for severe pain. Compare the two groups of patients' pain levels before and after the intervention. ⑤ Sleep quality: the Pittsburgh Sleep Index (PSQI) was used to evaluate the sleep quality of the two groups of patients. The higher the score, the worse the sleep quality.

### 2.7. Statistical Analysis

All data were entered using Epidata, and then, SPSS 25.0 was used for the statistical processing of the data. One-way ANOVA was used for measurement data expressed as mean ± standard deviation (*x̅*±*S*), and *χ*^2^ test was used for count data expressed as a percentage (%). Significant with statistical *P* < 0.05.

## 3. Results

### 3.1. General Data Analysis

There was no big difference between the two groups in female status, average age, course of the disease, degree of injury, and other general data by *t*-test and chi-square test (*P* > 0.05) (see Table 1).

### 3.2. Related Score Comparison

After nursing, the knee joint function score of the observation group was higher than that of the control group, while the postoperative pain, sleep quality, and anxiety self-rating scale scores were significantly lower than those of the control group. The difference was statistically significant (*P* < 0.05) (see Figure 1).

### 3.3. Nursing Quality Score Comparison

The scores for whole-process management, body position placement, risk assessment, rehabilitation training, all-weather service, system-wide management, and full-service after nursing in the two groups were significantly improved. The observation group was significantly higher than the control group. Statistics: this difference was significant for academic comparison (*P* < 0.05) (see Figure 2).

### 3.4. Nursing Effect Analysis

After nursing, the effective nursing rate of the observation group was 96.00%, which was significantly higher than that of the control group, which was 84.00%, and the difference was statistically significant by the chi-square test (*P* < 0.05) (see Figure 3).

## 4. Discussion

As healthcare costs continue to increase and patients' demands for health services increase, the health system surrounding conditions needs to continue to change and get better to meet new health challenges [17]. Early recovery after knee cartilage injury can reduce the knee joint tissue's serious physical or emotional harm response, can help increase in a good way the elimination of swelling, reduce pain, prevent stickiness/scar, and help increase in a good way the repair and healing of damaged tissue [18, 19]. In the usual nursing model, the focus of nurses' work is limited to mechanically executing doctors' orders, ignoring the mental feelings of patients [20]. Nursing model people-oriented, patient-centered nursing model puts forward the new nursing idea of 4F management [21]. In the nursing process, the mental and social well-thought-out and complete and thorough nursing are drawn attention to so that the patient's physical and mental fear and stress can be reduced, the after an operation quality of life can be improved, and the nursing quality can be improved, which truly reflects the nursing idea of 4F [22].

In this study, after nursing, the knee joint function score of the instance of watching, noticing, or making a statement group was higher than that of the control group, while the fear and stress self-rating scale score was much lower than that of the control group, suggesting that feedforward control combined with 4F management plays an important role in relieving patients' negative feelings of love, hate, fear, etc., and improving the quality of nursing. Chowdhury et al. [23] completed a knee joint function score to help improve the patient's knee combined function. Huang [24] studied the knee joint function score and fear and stress self-rating scale score after using a tiny camera surgery and effectively figured out the worth, amount, or quality of the patient's knee combined function and mental state. Knee combined harmful and angry behaviors can stop the patient's limb movement function, which is not good for their daily life and labor and increases their money-based heavy load and mental pressure [25]. Effective nursing actions that help in bad situations are needed to help patients with surgical treatment, to help increase in a good way the recovery of patients' knee and limb function, and to improve their after an operation repairing effects [26]. Feedforward control combined with 4F management combined with early repairing training action that helps a bad situation is under the combining in a way to make something better effect of pain relief actions that help bad situations combined with early repairing training measures to help increase in a good way the blood circulation of patients, reduce the surgical stress serious physical or emotional harm of patients, reduce the risk of poor outlook for patients, and quickly relieve after an operation pain in patients can improve the recovery of knee combined function [27].

In this study, the whole process management, postural placement, risk test/evaluation, repairing training, all-weather service, whole-system management, and all-around service of the two groups of patients were very much improved. The instance of watching, noticing or making a statement group was much higher than the control group, suggesting that feedforward control and 4F management measure something exactly The quality of nursing is better, and the quality of after an operation nursing of patients can be improved more complete and thorough and the event of risks can be prevented. As a viable management method, feedforward control is a crucial method to watch and evaluate the current status of patients, combine different things together, so they work as one unit of disease information, regularly describe a possible future event disease popular things ways things are going, and take serving to stop something bad before it happens actions that help bad situations [28]. According to all emergencies, patients and their families meet, communicate with them in advance to effectively reduce the risk, and compare other things complete supervising methods and nursing measures through a series of (reactions or responses to something returned information control measures [29]).

In this study, feedforward control combined with 4F management combined with early repairing training, through the creation and group of objects of an action that helps a bad situation group and training the team members on program-related knowledge, the nursing level of medical staff was improved, and patients were promised that something will definitely happen or that something will definitely work as described to receive producing a lot with very little waste nursing measures [30]. In thinking-related action that helps a bad situation for patients, by testing/evaluating the thinking-related shortage of patients with disease-related knowledge and giving corresponding education measures, improve the patient's thinking-related level, improve their self-management knowing about something and ability of disease pain and early repairing exercises, and improve their obedience of doctor's orders [31]. In pain management, pain evaluation of patients at different periods and corresponding nondrug and drug management measures can effectively relieve pain after the operation of patients [32–35]. In the early healing/repairing training, according to the after a physical operation condition of the patient, a series of targeted healing training programs are given to help increase in a good way the blood circulation of the tissue around the crack, reduce its swelling response, and speed up the recovery process of the affected limb [36–44]. Online pain management, guidance, and supervision of early healing training for patients are needed, and use of repairing evaluations and patient diaries [45]. Complete and thorough evaluation of the physical and mental health of the patients is carried out, and the action that helps a bad situation plan is appropriately improved according to the healing/repairing effect of the patients to significantly relieve the pain after the operation of the patients, improve their sleep quality, and improve the recovery of their knee combined function [46].

This study has some limits. First, the selected samples were all from patients who received nursing care or physical examination in our hospital, resulting in a certain degree of judging things based on opinions and preferences instead of facts included in something and when something is kept out or not included and related to large-area differences in the results of the study. Meniscal injuries are mostly found in the right knee, and the proportion of meniscal injuries in men is greater than that in women, and the incidence peaks between 20 and 29 years old. Rehabilitation care for patients of different ages was not provided in this study, and the effectiveness of this mode of care could not be demonstrated [47]. Finally, there were no in-depth study and long-term follow-up to understand the healing of patients with knee cartilage sports injuries after an operation.

In conclusion, feedforward control combined with 4F management combined with early healing training can effectively reduce knee cartilage sports injury fear and stress, pain after the operation, and sleep quality, improve after an operation quality of life, improve nursing quality, and help increase in a good way the recovery of knee combined function.

## Figures and Tables

**Figure 1:** Comparison of related scores (we used Epidata to input all data, and the nursing quality score was expressed as mean ± standard deviation. Chi-square test was used. After nursing, the knee joint function score of the observation group (Figure 1(b)) was higher than that of the control group, and postoperative pain (Figure 1(c)), sleep quality (Figure 1(d)), and anxiety self-rating scale score (Figure 1(a)) were significantly lower than those in the control group. Statistical *P* < 0.05, which was significant).

**Figure 2:** Comparison of nursing quality (we use Epidata to input all data, nursing quality scores are expressed as mean ± standard deviation, independent sample *t*-test is used, and the whole process management score, postural placement score, risk assessment score, rehabilitation training score, all-weather service score, system-wide score of the observation group, the management score, and full-service score were significantly higher than those of the control group, with statistical *P* < 0.05, which was significant).

**Figure 3:** Nursing effect analysis (We used Epidata to input all data, the nursing quality score was expressed as mean ± standard deviation, and the chi-square test was used. After nursing, the effective nursing rate of patients in the observation group was 96.00%, which was significantly higher than that in the control group, 84.00%, with a statistical *P* < 0.05, which was significant).

**Table 1:** Comparison of general data (*n*, (*x̅*±*s*)).

Group	Gender (men/women)	Average age (age)	Course of disease (year)	Degree of damage		
				I	II	III
Comparison group (50)	33/17	46.63 ± 10.32	3.31 ± 0.67	25	13	12
Observation group (50)	32/18	46.62 ± 10.31	3.33 ± 0.25	22	15	13
*χ* ^2^/*t*	0.044	0.005	-0.198	0.361	0.198	0.053
*P*	0.834	0.996	0.844	0.548	0.656	0.817

## Data Availability

No data were used to support this study.
